# Data Analysis of College English Speculative Reading Teaching Based on Multimodal Teaching Theory in a Complex Cross-Cultural Environment

This article has been retracted.

**DOI:** 10.1155/2022/1891937

**Published:** 2022-09-05

**Authors:** Tiantian Jiang

**Affiliations:** Business Foreign Languages Department, Shandong Foreign Trade Vocational College, Qingdao, Shandong 266100, China

## Abstract

With the continuous rise of my country's international status, the cultivation of students' cross-cultural thinking ability has become an important goal of college English teaching. Since the twentieth century, theories about critical thinking ability have been abundant, and how to improve students' critical thinking ability is also a hotspot of reform. In foreign countries, there are rich teaching models, but in China, it is still a major problem to be solved to cultivate students' speculative ability through specific teaching methods. How teachers' classroom teaching is related to the cultivation of speculative ability. In addition to having direct application significance for teachers to realize the cultivation of speculative ability in routine teaching, the research on these issues is conducive to opening the “black box” of classroom instruction. The most crucial tasks in teaching speculative reading and cross-cultural education in today's college English curriculum are the only means of enhancing students' critical thinking and cross-cultural communication skills. This paper analyses, researches, and applies the diagnostic evaluation model using data gathered during system usage. In order to enhance the diagnostic evaluation function of the college English diagnostic practice system and the associated test paper generation algorithm, the author then designs and implements two test recommendation algorithms in accordance with the diagnostic evaluation model.

## 1. Introduction

With the advancement of computer multimedia technology, words, images, sounds, and other media offer learners online learning opportunities that have never been possible before. Online learning has developed into a significant method of education and is a popular area of research in many universities and businesses both domestically and internationally [1]. It has also been made possible by big data and artificial intelligence technology [2, 3]. Helping students develop a thorough method of applying the language and autonomous learning is one of the goals of college English instruction. This will ultimately cultivate students' capacity for lifelong autonomous learning. Changing learners' ways of thinking is regarded as being of utmost importance in order to develop their capacity for lifelong learning and a sense of innovation. In order to develop the critical thinking skills of college English learners, this paper investigates the use of the four-resource model in reading instruction. The demand for international talent is growing daily, which necessitates the development of newer and more rigorous standards for college English teaching. Teaching English is essential for developing students' proficiency in the language as well as their capacity for problem-solving, critical thinking, and cross-cultural communication [4].

In this background, our country urgently needs a large number of talents with intercultural communication skills, and intercultural education has become the most important task in the teaching of English majors in colleges and universities [5]. Especially, the humanity of language determines that English learners can shoulder the important task of cross-cultural communication [6]. However, the actual college English teaching ignores the integration of language and culture, and the students' speculative and innovative ability to recognize, analyze, interpret and create the target language culture, which is not conducive to the students' mastery of cross-cultural knowledge, the development of cross-cultural communication and the improvement of their speculative and innovative ability [7]. It uses the technological achievements of scientific development to present the teaching process to users in the form of animation, which is interactive and authentic and can provide users with a realistic interactive environment and experience [8]. As this teaching strategy is improved, more and more barriers will be removed. While still offering instruction to every learner, the restrictions on time, location, and subject matter can be loosened [9]. The Internet has seen a considerable increase in the number of online learning platforms as a result of the recent, rapid development of various computer technologies [10]. These platforms have removed the limitations of paper-based learning materials, enabling more flexible and unconstrained online learning and practice.

Although the traditional teaching approach has greatly aided in the development of successive generations of human elites, it has gradually revealed some flaws that have become inescapable in the modern era: (1) the unequal distribution of educational resources causes a significant disparity in educational attainment between regions; (2) the one-to-many teaching approach forces teachers to concentrate their limited time and attention on a select group of exceptional students; (3) the lack of materials and potential dangers associated with scientific experimentation lead to a frequent abandonment of this method of learning; and (4) the uneven teaching abilities of teachers make the performance gap between students in related courses obvious. As science and technology have advanced, there has been a lot of interest in leveraging modern technology and the advantages of the Internet to address the issues with traditional schooling. But after utilizing these practice systems, it is not difficult to find out that their utilization is still limited to the traditional way of finishing questions and reading the answers, and that the feedback provided to students only focuses on the score, question answering, and question analysis. Teaching speculative English reading as a result became a component of cross-cultural education. In order to further open up a new situation in the teaching of speculative reading in college English for cross-cultural education, the author discusses his own understanding and opinions based on his thinking experience and work perception of theoretical learning over the years. He does this with an eye toward in-depth exchanges with colleagues.

As a result, the author believes that given the lack of diagnostic evaluation in online learning platforms, real data collected in the system should be processed and studied using current, widely used data mining and machine learning technologies. Following this, a diagnostic evaluation model for college English should be developed, and a customized and targeted recommendation algorithm for test questions should then be presented.

## 2. Related Work

A thorough comprehension of the text is what speculative reading instruction entails. It includes paraphrasing and evaluation skills that help readers distinguish between relevant and irrelevant facts and opinions, as well as identify the author's purpose and tone. It also includes reasoning skills that help readers infer implications, fill in the gaps in the information, and reach logical conclusions.

In the summary of research on special topic teaching of college English, Hardison combed the academic circles' three different understandings of English as defined by “special topic teaching,” three views of English as a theoretical basis, and the different integration patterns based on textbooks and elective courses [11]. Satar and Wigham By comparing English special-topic teaching with unit teaching and single-part teaching, several essential elements of English special-topic teaching are obtained: (1) according to the perspectives of works, writers, themes, and students, “gather articles into categories”; (2) problem situations; (3) teaching tasks are more open, closer to life, and pay more attention to the cultivation of students' abilities; and (4) teaching process is the thinking construction process of students' learning [12]. Peng explained the cohesion, openness, comprehensiveness, inquiry, practicality, and other characteristics of thematic learning in her master's thesis. Her dissertation “research on the current situation and strategies of college English special teaching” expounds on the principles of highlighting research-based learning methods in college English special teaching, realizing modular learning, and expanding curriculum resources based on textbooks [13]. Querol‒Julián and Fortanet‒Gómez put forward the implementation ideas of special subject teaching in university from three aspects: material selection, sequence, transformation, generation, integration, and improvement, and illustrated the basic process of module teaching with video lessons: self-reading-reading-reading-reading-writing [14]. Chris believes that the university teaching methods include: methods that are suitable for the process of teaching cognition, methods that are suitable for students' cognitive independence, and intellectual ways and methods in teaching cognition activities [15]. and Andrew [16] According to the unified standard of teaching forms and methods, the basic teaching methods of colleges and universities are divided into English categories: (1) classroom teaching methods: including lecture, experiment, and discussion; (2) self-study and self-study guidance methods: including reading guidance, review, homework, and counseling; (3) on-site teaching methods: including visiting method, investigation method, practice method; and (4) methods of scientific research training: including usual scientific research training, thesis, and design. From the perspective of teaching tasks and characteristics, Wang J divides college teaching methods into the following: (1) theoretical teaching methods, such as teaching method, conversation method, and demonstration method; (2) explore teaching methods, such as discovery method, self-study method, and discussion method; and (3) practical teaching methods, such as visiting method, practice method, and experimental method, [17]. Tuero's research on college English teaching methods shows that the new English teaching concept has been produced, but it has not been implemented in English teaching practice, and the traditional teaching methods that are not conducive to cultivating students' ability still account for a large proportion. Teachers' guidance for students in English learning methods and practice methods is insufficient, and college English teachers have no research awareness of teaching methods, etc. [18]. The current teaching concept of college English classrooms in China is outdated, the teaching content is out of touch with the actual application of English, and the amount of teaching information is small. The reform of college English teaching methods should be carried out through the following points: using “case teaching method” to introduce English concepts, “comparison method” to introduce concept comparison, “problem-driven method” to carry out discussion classes, English modeling ideas in the classroom, etc., [19]. The research on TN shows that teachers and students in universities in China have low expectations for effective teaching methods, insufficient awareness of the importance of teaching methods, and inadequate measures to improve teachers' and students' teaching methods literacy in universities [20].

To sum up, we can see that the current research on undergraduate classroom teaching methods in my country is still mostly speculative research, and there is little evidence for empirical research. Scholars and educators in our country have noticed the importance of university teaching methods, but on the other hand, the actual application of teaching methods has not changed much and basically continues the traditional teaching methods. Why does this happen? Next, we will explain the reasons why the teaching methods are outdated and difficult to use in innovation.

## 3. Methodology

### 3.1. Data Mining Combined with English Speculative Reading Teaching for Analysis

In recent years, data mining has captured the interest of the vast majority of scientists, who are eager to convert a large amount of disorganized data into knowledge and information. This research will also investigate the question association rules using data mining. Data processing and analysis are used in a process called “data mining” to find previously unknown information in collections of unordered data. The college English diagnostic practice system also has this problem. The practice and confirmation of the specifics of the results are the two main goals of the current diagnostic practice method for college English learners. The practice functions contain six alternative test grouping algorithms: the four-level real exam practice, random test question grouping, grouping by question type, category of knowledge points, maximization of knowledge points, and grouping by knowledge point association criteria. Speculative reading teaching is a series of teaching activities in which teachers teach students how to carry out speculative reading. It is a high-level understanding of teaching materials and articles, including the skills of article interpretation and content evaluation. The purpose is to help students distinguish between important and nonimportant information, facts, and views. Different languages have different cultures, and different cultures have different habits and characteristics. English culture has its distinctive uniqueness and nationality, which is a typical symbol of national differences. The purpose of learning English is to understand and master English culture, and then to realize effective communication and exchange with people of English-speaking nations or countries. One is to be proficient in English language knowledge, application skills, and learning strategies. The second is to cultivate superb cross-cultural thinking ability, able to accurately understand and use English for cross-cultural communication. Once college students have excellent cross-cultural thinking ability, they can better understand and master the intention of the communication object, so they have a very favorable competitive position in English services. With the development of globalization and diversification in the world, China has become more and more influential in politics and the economy on the world stage. At this time, English is no longer a simple major or course, but an important means to improve students' international competitiveness. Under this background, intercultural English teaching can cultivate more intercultural talents. The highest level for college students to learn English is to learn to think in English, expand their thinking ability and improve their comprehensive English quality. The speculative reading teaching not only cultivates students' speculative ability but also virtually broadens students' thinking horizon, promotes the improvement of their overall thinking ability and then drives the overall improvement of English comprehensive quality.

There are six distinct categories of data mining tasks: association analysis, cluster analysis, classification, prediction, time-series patterns, and deviation analysis. The algorithm flow of data mining in English reading and critical thinking teaching is as follows: (1) Text data collection. Identifying data sources and obtaining corpus are generally the first steps of text data mining. At present, the required data are usually obtained in the form of grabbing network data. (2) Data preprocessing. Due to a large number of online comments and unstructured data, the comment data collected by web crawler technology can generally meet the needs of quantity and topic relevance, but it cannot make the initial data machine readable. (3) Text feature mining. This is the main link in the process of data mining. Using a neural network, machine learning, data analysis, and other related technologies, we can mine the key elements such as product features, comment opinions, and user emotions implied in the review text, and realize the classification, clustering, and correlation analysis of the text topics. (4) Display of visual results. Usually, visualization tools are used to display the data analysis results in graphs, charts or interfaces, highlighting the value of data, making the data results easier to communicate, more vivid and friendly, and more intuitive to feel the key information conveyed by the research results.

“Speculative expression” is an activity that takes place in “speculative reading” and covers the beginning and end of reading. The essential level analysis of “speculative expression” can be completed in speculative reading, focusing on the accumulation of learners' thinking ability and expression skills. For example, in speculative reading, students can analyze and demonstrate current affairs comments, and comprehensively carry out speculative discussions and debates around key topics. Based on the above analysis, the “critical reading and expression” studied in this paper is a process that takes the construction of learning task groups as the core carrier and critical thinking as the learning method, so as to continuously improve students' critical thinking ability and cognitive depth in reading and writing teaching. No matter “reading” or “expressing,” we should focus on “thinking.”

### 3.2. Optimal Design of Speculative Reading Based on Data Mining

In order to understand the implementation mode of “critical reading and expression” learning task group more intuitively and clearly, this paper designs different forms of teaching activities combined with relevant concepts in the research process. The effective carrier of learning task group can play an important role in the process of critical reading and expression teaching, and the two promote each other. With the help of learning task group, critical reading and expression can be guided, and critical reading can be more reasonable and efficient to promote the construction of learning task groups. First, the teaching mode of learning task group can effectively improve students' logical thinking ability and the application level of critical thinking, improve students' reading and writing skills, thinking ability, and effectively improve the pertinence and effectiveness of teaching activities. Second, the implementation of speculative reading and expression requires a reasonable design of learning task groups, and the acquisition of reading and expression needs to be integrated. The revision group of general English curriculum standards pointed out that “teachers should carry out project-based teaching design around speculative learning.”

It shows that the educational activities driven by this goal and task, that is, listening, speaking, reading, and writing, have more practical significance, can carry out teacher-student dialogue and student-student dialogue in specific situations, can improve the critical thinking ability, and can realize the organic combination of problem topics, reading appreciation, project guidance, combing and inquiry, expression and communication, so as to improve critical thinking, improve thinking and guide the design of learning task groups. Speculative reading includes three learning contents: “first, understanding the author's attitude, viewpoint and language features; the second is to analyze the logic and method of the author's point of view; and the third is to demonstrate and evaluate the ideological value of the text and make a correct judgment.”

One of the most popular machine learning algorithms is the decision tree algorithm. It involves classifying or regressing data using a variety of operating rules. Regression and classification decision trees are two different types of decision trees. Regression decision trees perform regression calculations on continuous variables, while classification decision trees classify discrete variables.  Figure 1 depicts a decision tree as an illustration.

Decision tree algorithm finds the possible classification or regression rules in the data by constructing the data structure of tree. The core of decision tree algorithm is to ensure that the constructed decision tree must have the characteristics of accuracy and small scale. The construction of decision tree can be divided into two steps. First, the generation of decision tree: the data set to be trained needs to be divided into decision trees. The second is pruning the decision tree. Use pruning technology to test the decision tree generated in the previous step, mainly use the validation set to test the classification and regression rules of the decision tree, and delete those branches that affect the accuracy. Six components make up the English thinking model: thinking purpose, thinking process, thinking material, self-regulation, thinking quality, and noncognitive and cognitive factors. The beauty of this model is that it puts self-regulation at the apex, which is metathinking. As shown in Figure 2.

The construction of decision tree can be divided into two steps. The first is the generation of decision tree: the data set to be trained needs to be divided into decision trees. The second is to prune the decision tree: use pruning technology to detect the decision tree generated in the previous step, mainly using the validation set to test the classification and regression rules of the decision tree, and delete those branches that affect the accuracy. The steps of decision tree algorithm are as follows: (1) starting with a single node of the training set; (2) if all attributes belong to a set, mark the tree node to make it a leaf; (3) otherwise, the algorithm will select the attribute with the strongest classification ability as the current node of the tree; (4) the training will be divided into many subsets according to the difference of the attribute value of the node currently to be divided, and each attribute value is divided into a branch. For the subset obtained in the previous steps, the previous steps are recursively executed to construct a decision tree; and (5) all samples to be trained are divided into the same category; all attributes have been used in dividing the samples; if in a certain In the branch, if the samples that have already been classified are not included, the samples with a larger number are divided into a leaf.

When selecting attributes to divide, C4.5 algorithm uses information gain rate to consider, which avoids the defect of selecting attributes with more values when using information gain. The definition formula of information gain rate is as follows:

(1) $$\begin{array}{c} \text{GainRatio}\left(A\right)=\frac{\text{Gain}\left(A\right)}{\text{AplitInfo}\left(A\right)}, \end{array}$$

where gain (a) is the information gain, and its formula is as follows:

(2) GainA=InfoD−InfoDA.

Split info (a) is the split information value, and its formula is as follows:

(3) $$\begin{array}{c} {\text{SplitInfo}}_{A}\left(D\right)=-\sum_{j=1}^{V}\frac{\left|D_{j}\right|}{\left|D\right|}\times \;\log_{2}\left(\frac{\left|D_{j}\right|}{\left|D\right|}\right). \end{array}$$

The decision tree algorithm has the advantages of high classification accuracy, simple algorithm generation, antinoise data, good robustness, etc., and has been widely researched and explored by researchers in the field of machine learning.

Carrying out cross-cultural English speculative reading teaching is essentially an educational and teaching reform. To effectively do this teaching work, we must carry out in-depth teaching and scientific research activities. First, we should change the teaching methods, actively carry out independent inquiry teaching, and effectively stimulate students' learning desire and enthusiasm. In classroom teaching, one-sided emphasis is placed on the memorization and use of words and grammar, while the in-depth understanding, communication, and criticism of cross-cultural education are ignored. In this way, although students know the customs and cultures of English-speaking countries through teachers' indoctrination, they lack a deep understanding of their cultures. At present, although many scholars and teachers have studied cross-cultural speculative reading teaching, the school leadership and management have not paid enough attention to it, which makes these studies lack due to effect.

### 3.3. English Speculative Model Based on Learning State Algorithm

The construction of a logical thinking scaffold needs to accurately state the textual information, including the relationship between conditions and conclusions, which is the basic way to strengthen the understanding and communication of viewpoints and form rational judgments by means of stating viewpoints. In the process of expressing or analyzing their views, it is necessary to pay attention to the establishment of logical thinking, to improve the adequacy, rationality, and inevitability of factual statements or textual information statements, and to avoid mistakes between sufficiency and necessity. Rigorous argumentation needs to be analyzed with the help of scientific derivation and causal inference, covering the judgment and reasoning knowledge of various formal logical thinking. Logical reasoning methods cover a variety of methods, which are similar to the demonstration methods commonly used in Chinese teaching. All kinds of “exemplification” analysis cover reasoning and other contents. It is necessary to explore new arguments from various typical cases, summarize and reason various cases and prove arguments. From the perspectives of “explanation and analysis, evaluation and reasoning, explanation and self-regulation,” we can cultivate students' cognitive skills in critical thinking. Critical thinking takes the following of cognitive process as the main premise, and evaluation and analysis include multiple stages, the first stage is questioning. The second stage is thrust evaluation, which means that in order to achieve the purpose of a comprehensive evaluation, a verification must be carried out on the basis of the previous stage. The third stage is to explain the verification process and make some amendments to the verification results.

In order to give learners individualized guidance, the learning state evaluation algorithm primarily calculates learners' mastery of knowledge points and questions, learners' attention coefficient, and learners' learning type. The following actions are detailed:

(1) Read the knowledge points of the students and the question type scoring rate. Read the students' knowledge points and the question type scoring rates from the database, and store them as a matrix. There are n learners, and each learner receives M items worth of knowledge points and questions. The element *x*_*ij*_ in the matrix indicates the score rate *J* of the *i*th learner. The formula of the matrix is as follows:
  (4) $$\begin{array}{c} \left[x_{ij}\right]=\left[\begin{array}{ccc} x_{11} & x_{12} & x_{1m}\\ x_{21} & x_{22} & x_{2m}\\ x_{n1} & x_{n1} & x_{nm} \end{array}\right]. \end{array}$$
(2) Processing continuous data
The learning state evaluation algorithm can only process binary data, therefore even though the knowledge points and question scores are distributed as decimals with a range of [0, 1], these data must be processed. The average value of each knowledge point and the scoring percentage for each question type is used to determine the threshold, which is also the benchmark for judging whether mastery has been attained. If the judgment is more than or equal to the threshold, it is considered to have been mastered and given a mark of 1, otherwise, it is not mastered and given a mark of 0. The calculating formula is as follows:
  (5) $$\begin{array}{c} \text{Line}\left(x_{ij}\right)=\left\{\begin{array}{c} 0,x<\frac{\sum_{i=1}^{n}x_{ij}}{n}\\ 1,x\geq \frac{\sum_{i=1}^{n}x_{ij}}{n} \end{array}\right). \end{array}$$
(3) S–P table row and column calculation
Suppose *x*_*ij*_ is the scoring rate of the knowledge point of type *j* of the *i*th learner, then the sum of the scores of learner *i* is the sum of the number of correct answerers of the type *j* of the *x*_*i*_ knowledge point; The formula is as follows:
  (6) $$\begin{array}{c} x_{i}=\sum_{j=1}^{m}x_{ij}. \end{array}$$
(4) Calculate the mastery of the learner's question type knowledge points and the learner's attention coefficient
Let *x*_*ij*_ be the scoring rate of the knowledge point of *J*-type question of the *i*th learner, *x*_*i*_ be the total score of learner *I*, *x*_*j*_ be the sum of the number of correct answers of knowledge point *J*, *μ* Is the average score rate of learners, then the simplified calculation formula of learners' attention coefficient CSI is as follows:
  (7) CS=i1−∑j=1nxijxj−xiμ∑j=1xixj−xiμ.
(5) Determine the type of learners.
Determine the learners' mastery and attention coefficients using the classification criteria for learners' types.
(6) Output results
Output learner's knowledge point question type scoring rate, learner's attention coefficient, and learner type. To sum up, the above are the specific steps of the learning state evaluation algorithm, and the flowchart is shown in Figure 3.

If there is a considerable difference between the maximum and minimum values in the data set, the RMSE will be dominated by certain bigger values. Even if many smaller values are accurately predicted, this will lead to a large RMSE since some bigger values are not correctly anticipated. In the event that the prediction of certain smaller values deviates from reality, RMSE may be lower than it was previously. This problem can be solved using RMSE by first taking the logarithms of the actual value and the anticipated value, then solving them. RMSE and RMSLE are calculated as follows:

(8) $$\begin{array}{c} \text{RMSE}=\sqrt{\frac{\sum_{i=1}^{n}{\left(X_{obs,i}-X_{\mathrm{mod}\text{el},i}\right)}^{2}}{n}},\\ \text{RMSLE}=\sqrt{\frac{1}{n}\sum_{i=1}^{n}{\left(\log\left(X_{obs,i}+1\right)-\log\left(X_{\mathrm{mod}\text{el},i}+1\right)\right)}^{2}}. \end{array}$$

Among them, *X*_*obs*,*i*_ is the predicted value and *X*_model,*i*_ is the true head value.

The design of database should not only meet the needs of users, but also reduce the redundancy of data as much as possible, reduce the dependence between data as much as possible, separate them, and require the database structure to fully meet the output and input of various information. Considering merging association rules *R*1 and *R*2, there may be two rules with the same or similar left and right parts, or the left or right parts of the two rules can be merged, or their support and confidence differences are very small. For the case that the attributes on the left and right sides of the two rules are the same and the attribute values are similar, we can consider merging the two rules into one, (URL = 2.2, 20 < study time < 40), then the formula for calculating the support of the new rule *r* according to rules *R*1 and *R*2 is as follows:

(9) $$\begin{array}{c} \text{S}\left(r\right)=\frac{\text{s}\left(r_{1}\right)\times \text{dbsiZe}\left(r_{1}\right)+\text{s}\left(r_{2}\right)\times \text{dbsize}\left(r_{2}\right)}{\text{db\_size}\left(r_{2}\right)+\text{db\_size}\left(r_{1}\right)}. \end{array}$$

The calculation formula of support degree on the left side of the new rule is as:

(10) $$\begin{array}{c} S\_1\text{hs}\left(r\right)=\frac{\text{s\_lhs}\left(r_{1}\right)\times \text{db\_size}\left(r_{1}\right)+\text{s\_lhs}\left(r_{2}\right)\times \text{db\_size}\left(r_{2}\right)}{\text{db\_side}\left(r_{2}\right)+\text{db\_size}\left(r_{1}\right)}. \end{array}$$

The formula for calculating the confidence of the new rule *R* according to the rules *R* and *R* is as follows:

(11) $$\begin{array}{c} \text{confidence}\left(r\right)=\frac{s\left(r\right)}{s\_1hs\left(r_{1}\right)}. \end{array}$$

Although module teaching still needs further research in practical operation, it is student-oriented, advocates the openness of learning resources and the exploratory nature of the learning process, provides a broad space for personal development, and promotes the construction of innovative talents. The concept of lifelong education is of great significance. It is also an important theoretical framework for our curriculum reform. To sum up, it can be seen that the student subjectivity, speculative reading and writing, reading and writing integration, and resource integration contained in the teaching design of the special topic “speculative reading and expression” have a deep theoretical foundation. These theories are still valued by the educational circles in the inheritance and reform, which shows that they have the value and possibility of implementation.

## 4. Result Analysis and Discussion

As the learning task group of “Critical Reading and Expression” was just put forward in 2017, its teaching method is quite different from traditional teaching, there is no fixed implementation mode, and the specific implementation varies greatly among different regions and schools. The current research shows that the academic community is paying more and more attention to the impact of this task group on the development and improvement of students' thinking. Therefore, the author intends to investigate whether the teaching of “speculative reading and expression” has been implemented in high school in Xiamen and whether it has been explored. Good teaching cases and what are the main reasons that currently hinder teaching attempts. This method is mainly used to understand the front-line teachers' understanding of “speculative reading and expression,” the current situation of teaching implementation, practical difficulties, and their own teaching suggestions. Among them, 15 front-line teachers with rich teaching experience who have taught in a city for more than 5 years were contacted. The questionnaire is divided into two parts: the student questionnaire and the teacher interview questionnaire. In order to show the contents of the questionnaire more intuitively, the author will elaborate on the ideas of questionnaire design in Tables 1 and 2 in the form of tables mentioned below.

Three moderately difficult questions are arranged here keeping in mind that they should not take up too much of the students' study time and their general cognitive level. The three questions are all taken from sample test papers of speculative teaching experts in order to increase the scientific nature of the test results. These questions are also based on the students' prior learning experiences and do not go beyond their acceptable range.  Table 2 shows that the majority of students received scores for the diagnostic evaluation, learning state evaluation, knowledge point diagnosis, and question type diagnosis that were greater than or equal to 3 points, with an average score of more than 3.6 points for each evaluation. The user's score, which is visible to be between general and satisfactory and tends to be satisfactory, demonstrates to some extent the diagnostic effect of the diagnostic evaluation model.

In addition, the author also collected the practice data of the students in this experimental class using the diagnostic practice system and used the CET-4 score prediction model to predict the scores. The comparison between the predicted values and their real values in this CET-4 test is shown in Figure 4, with the scores of CET-4 on the ordinate.

As can be seen from Figure 4, there is little difference between the predicted value of grade 4 scores and the actual value of the students in the experimental class, the predicted value is relatively accurate, and the RMSE between the actual value and the predicted value obtained through calculation is 19.546, The RMSLE is 0.121, also very close to the previous data.

The bar chart reveals that the overall level of students' critical thinking ability has improved. Generally speaking, the percentage of all subaspects of weak students' critical thinking ability has decreased, and the number of excellent and excellent students has increased. Among the five subaspects of critical thinking ability, reasoning and analysis ability have changed greatly. The weak level students have decreased from 28% to 31% to 12% and 15%, both of which have decreased by 15 percentage points, while the strong level students have increased by 10 percentage points and the corresponding 7% (from 9% to 15% to 19% and 22%). Compared with other aspects, the assessment ability fluctuates from 23% to 20%, that is, only 3% of students have made progress in this regard for the intervention of reading teaching. As shown in Figure 5.

During the semester, the authors designed five reading tests and recorded scores on all tests. The table below shows the average of each quiz during the last quiz is the average of all five quizzes. Two groups represent two people and each class has 55 students. It should be emphasized again that the full score for each quiz is 16, as shown in Table 3 and Figure 6.

I compared the experimental time with NOBOOK and OpenGL in order to confirm the effectiveness of the suggested framework. In addition, I implemented single-mode (gesture) interaction (sive) on the virtual experimental system set up in this paper in order to minimize the impact of various systems. Twenty individuals were invited to take part in acid-base verification tests on various testing grounds.  Figure 7 shows the total amount of time required to complete the acid-base detection experiments using various methods, including the time required for user adaptation, trial and error, questions, and experiment understanding.

The findings demonstrated that as the number of experiments increased, the experimental time gradually decreased before gradually stabilizing in the final three experiments. Data analysis reveals that mouse interaction is very effective at cutting down on time consumption. The time cost of miivep, however, gradually catches up to that of NOBOOK and OpenGL based on mouse interaction as the number of experiments rises, demonstrating that miivep can also be comparable to mouse interaction in terms of time consumption while offering a more natural means of interaction. According to the experimenter's feedback, SIVE only offers a single mode of interaction, which users must spend time getting used to and remembering, whereas multimodal interaction better accommodates different users' interaction habits and allows each user to interact smoothly according to his or her own habits.

The system performance of MI-VE based on MMIP is assessed using VEES. Some scoring indicators are appropriate for conventional teaching experiments because the VEES score is designed for the virtual experiment system (such as robustness). Each indicator receives a score of 100 points. Then, we asked ten middle school teachers to rate various VEES indicators of conventional experimental teaching and VR experimental teaching, and the average result was used to determine each indicator's final score, as shown in Figure 8.

In Figure 8, each number represents 1-experience authenticity, 2-effect authenticity, 3-organizational difficulty, 4-safety, 5-learning effect, 6-equipment vulnerability, 7-explorability, 8-learning speed, 9-repeatability, 10 sufficient experimental materials, 11 teacher concentration, 12 robustness. In traditional experimental teaching, the easy damage of equipment is a serious problem, and the lowest score is obtained. VR lab still has an obvious disadvantage: lack of explorability. VR lab is only a virtual system that simulates real experiments, and cannot really realize the randomness and contingency of experiments. Users' experiments are just reproduction rather than exploration and discovery. In addition, the unique attributes of VR-Lab are experienced authenticity and phenomenon authenticity, but obviously, teachers think that these two items do not perform well on VR-Lab. These are the two points that the virtual experiment system lacks and needs to be improved most, and they are also the problems that researchers need to solve urgently. The requirement analysis of the diagnostic evaluation subsystem is carried out, and the user requirements and interface design of the system are mainly explored. The author chooses the technical framework that will be employed by the system based on the demand analysis. An external interface is used to generate the diagnostic evaluation module, which is then recorded in the system database for users to access. The diagnostic practice system for college English will include a test-setting module. The author creates the operation process and associated database tables for the subsystem in accordance with the aforementioned demand analysis and technical scheme and implements all of the diagnostic evaluation subsystem's functions in accordance with the system design and technical scheme. The college English diagnostic exercise system is now complete with the addition of the diagnostic evaluation subsystem.

## 5. Conclusions

Judging from the current situation, if we want to improve the effectiveness of English teaching, we must improve students' learning depth, vigorously carry out independent inquiry learning, and turn students' passive learning into active exploration and discovery. Teachers should strengthen guidance and allow students to analyze and evaluate foreign cultures objectively and rationally. It is necessary to appropriately organize and carry out some high-level cultural seminars, guide students to improve their knowledge and understanding of the learning content in the exchange, and convert the teaching content into practical experience, so as to improve their cross-cultural thinking ability. First, we should increase the assessment contents and standards of cross-cultural education and speculative reading teaching, stimulate teachers' enthusiasm to actively carry out cross-cultural education and speculative reading teaching, and stimulate students to establish scientific cross-cultural awareness and speculative awareness; Second, we should improve the reward and punishment mechanism, stimulate teachers' desire for innovation and enthusiasm, and stimulate students' interest and enthusiasm in creative learning through strong assessment, reward, and punishment. This study aims to find an effective and feasible method to cultivate college students' communicative competence in English teaching.

## Figures and Tables

**Figure 1:** Decision tree legend.

**Figure 2:** Thinking pattern diagram.

**Figure 3:** Flow chart of learning state evaluation algorithm.

**Figure 4:** The ordinate is a four-grade fractional graph.

**Figure 5:** Statistical description of the variation of five dimensions of critical thinking ability.

**Figure 6:** Comparison of predicted and actual values.

**Figure 7:** Comparison of the time spent in the experiment.

**Figure 8:** VEES score.

**Table 1:** Contents of student questionnaire.

Title serial number	Survey content	
Question 1	A survey of students' current speculative level	Students' judgment of “assumption premise”
Question 2		Students' understanding of “arguments”
Question 3		Students understand the situation of memorizing stories
Question 4	Students' reading habits and cognition	Students' reading tendency
Question 5		Students' understanding of secretaries with “critical thinking”
Question 6		Students' preference for interpreting speculative texts
Question 7	Students' attitude towards authority	Students' attitude towards famous sayings
Question 8		Students' attitude towards hot information on the internet
Question 9		Students' attitude towards book knowledge and teachers' personal profile

**Table 2:** Contents of teacher interview questionnaire.

Title serial number	Survey content	
Question 1	Title serial number	Understanding of “critical reading and expression”
Question 2		Has the “critical reading and expression” task group been taught?
Question 3		Guidance to students in reading teaching
Question 4	Teachers' teaching practice	Teaching guidance for students' writing
Question 5		The usual reading habits
Question 6		Do you have a debate on sun's topic
Question 7	Teachers' teaching problems and suggestions	Problems in the teaching of “critical reading and expression”
Question 8		My own thoughts on implementing students' thinking learning

**Table 3:** Average score of reading test.

No/group	1	2	3	4	5	Mean
1 (experimental)	9.42	9.41	10.64	14.3	12.46	11.43
2 (control)	9.16	7.61	8.12	10.6	9.14	8.12

## Data Availability

The data used to support the findings of this study are available from the author upon request.
